This article has been retracted.

# Application of Lightweight Deep Learning Model in Vocal Music Education in Higher Institutions

**DOI:** 10.1155/2022/6757341

**Published:** 2022-03-26

**Authors:** Zhen Zhu, Zhongqiu Xu, Jing Liu

**Affiliations:** ^1^Ukrainian National Tchaikovsky Academy of Music, Kyiv 999146, Ukraine; ^2^Guangzhou Sport University, Guangzhou, China

## Abstract

The aim is to improve the teaching quality of music majors and cultivate their innovative ability. This article takes Vocal Music Education (VME) method as the research object to explore the teaching reform of Music Major courses. Firstly, this article makes an in-depth study on Big Data Analytics (BDA) and Digital Twins (DTs) technology and constructs a DTs platform connecting real teaching space and virtual teaching space. Secondly, the DTs platform is divided into online learning feature analysis and virtual-real teaching space integration functional modules. This article explores the online immersive education process design and technology application of the DTs platform from the two aspects of teaching and technology. Afterward, it designs a student action and expression recognition network based on the Visual Geometry Group (VGG) Net model and Google Net model in teaching data collection and management. Finally, the proposed system is tested. The test results show that the active and passive interaction curves of the traditional VME system have no obvious fluctuation, indicating that the interaction of the traditional VME system is not strong, and the ability of active feedback information is poor. By contrast, the active and passive interaction curves in the proposed VME have large fluctuations, showing that the proposed VME has more frequent interaction, and the teaching information can get real-time and active feedback. Therefore, the proposed VME system can better stimulate students' learning desire. Meanwhile, the constructed Neural Network (NN) has the highest recognition accuracy of 99.07% on the student action and expression dataset. When tested with the image data taken by the research experiment, the highest accuracy is 89%, with an average of more than 85%. The proposed VME system provides ideas for applying DTs technology in the college of music education.

## 1. Introduction

Vocal Music Education (VME) is a human activity to continue the aesthetic concept of vocal music and the content, skills, and creative singing methods. VME can be understood from either a broad sense or a narrow sense. In a narrow sense, there is a clear relationship between teachers and students, teaching time, teaching place, determined teaching content, and targeted teaching activities. There is no clear relationship between teachers and students and teaching intention in a broad sense. Still, objectively speaking, it impacts people's vocal music aesthetic concept, vocal music art cultivation, and vocal skills. VME is an important part of music teaching in higher institutions and a complex and systematic teaching project. It shoulders the important tasks of training vocal music professionals and technical talents, training middle school music teachers, and improving students' comprehensive music quality. Meanwhile, VME is different from the education of other music disciplines, which is a very abstract education and not intuitive except for the external singing performance. Therefore, people deem VME the most challenging musical course in higher institutions [1, 2]. Particularly, VME in Chinese higher institutions has gone through four periods: germination period, development period, slow period, and climax period. Specifically, the development period has seen the introduction of many professional teachers into higher institutions, who have a rapidly increasing teaching level. At the same time, there are also teachers with good teaching levels in relevant institutions. In the climax period, the overall feature of VME is the common development of Bel Canto and national singing. Especially in the 1980s and 1990s, Chinese vocal music students and actors have presented themselves on the international stage. The singing level of Chinese national and local style works has improved rapidly. These facts prove that China's VME has made great achievements and rapid progress. Chinese Bel Canto is in line with the world smoothly, and the “Chinese vocal music school” with the perfect combination of Bel Canto and national singing has begun to take shape. With the rapid development of new technologies, “big data + Artificial Intelligence (AI)” has become a new driving force and way of thinking in modern society. On the other hand, Digital Twins (DTs), a new technology that can effectively realize the intelligent interconnection and interactive integration between the material world and the information world, come into being. Consequently, a DTs platform connecting real teaching space and virtual teaching space can be constructed, which has become the “digital artery” of network teaching space. The digital platform utilizes technological modules, such as online learning feature analysis and virtual reality (VR) teaching space integration and analysis. Through the deep integration, mapping, and mirroring of teaching and learning (TLT) network, new digital productivity can be injected into immersive online teaching [3, 4].

Researchers have also done a lot of research in music teaching in higher institutions. Wacker [5] explored the views of music education major students on curriculum planning in college courses. Cheng et al. [6] argued that music and natural language share many basic processing mechanisms. They evaluated the effectiveness of cultivating music majors' autonomous learning in performance practice through a series of curriculum reforms. Martin Gutierrez et al. [7] contended that applying multimedia promoted application research and retrieving specific information from a large number of music-related data had become a challenge in music information retrieval. A multimode end-to-end Deep Learning (DL) architecture HitMusicNet was proposed to predict the popularity of music recording. Molero et al. [8] helped students learn music by designing a new method based on Mixed Reality (MR) and games to stimulate students' interest in learning. As a result, students' learning motivation improved, and their performance of music style was roughly understood. Cai [9] explored the application of the DL algorithm in music arrangement and composition and the role of blockchain in digital music copyright protection. Firstly, a single tone melody composition model based on deep Generative Adversarial Networks (GANs) was constructed, and the synthesis performance of the model was analyzed with the hymn as the input sample. On this basis, a multi-instrument collaborative arrangement model based on multitask learning was proposed, and its composition performance was analyzed with the actual music as the input sample. Finally, an improved Practical Byzantine Fault-Tolerant (PBFT) algorithm was proposed, and a digital music copyright protection system based on blockchain was designed. The results showed that the accuracy of deep GAN in predicting soprano and alto melodies was 2.29% and 3.32% higher than that of the DeepBatch model, respectively. The multi-instrument collaborative arrangement model based on multitask learning was superior to other models in harmony score, note accuracy, Levenshtein similarity, Mean Square Error (MSE) of note distribution, null value, and convergence speed. In 2006, the top academic journal “Science” published an article on DL, a pioneering achievement in the DL field, and had since established Hinton's authority in the DL field. Zhang [10] designed an electronic music recognition model based on Convolutional Neural Networks (CNNs), took the electronic music spectrum waveform as the input, and extracted the input images using the mixing and sampling method of multilayer feature fusion. Then, they trained the CNN by the backpropagation (BP) algorithm and piloted the electronic music classification and recognition through the SoftMax classifier. The experimental results proved that the designed model could effectively remove the noise in electronic music. When the number of iterations reached 100, the model fitting error could reduce to the lower limit, and the average recognition rate was about 98.5%. Xw and Yao [11] used Neural Network (NN) to teach students music and verified the examination process of students' music courses after learning.

To sum up, there are still some problems in VEM in Chinese higher institutions. (I) VME has high professional and technical requirements. Educators are also troubled that vocal music is challenging to learn and teach. The reason is that the vocal music teaching process is not a simple imitation learning but to control the body through the perception and understanding of ideology. (II) For a long time, only some simple musical instruments have been used in teaching props in VME. With the continuous development of science and technology, electronic teaching equipment has been more frequently seen in the classroom, but the traditional teaching modes still prevail in substantive teaching. The emergence of the intelligent economy brings a provocative social change. The current educational sector has gradually become a practical field of real-time interaction and integration of virtual and reality. DTs have the technical characteristics of virtual reality symbiosis, high virtual simulation, and high real-time interaction. Its application trend also extends and expands from the industrial field to education, among many others. The application of DTs in the education field is mainly reflected in several aspects. 1. It is a visual tool to help Science, Technology, Engineering, Mathematics (STEM) education, maker, and innovation education. 2. As a historical data collection and analysis platform, DTs optimize teaching evaluation and promote educational equity as a distance education platform. 3. DTs promote cultural and historical education as a means of cultural heritage reproduction. 4. DT is a communication platform connecting formal and informal learning. With the emergence and application of DTs classroom and DTs campus, DTs will further promote education reform by intelligent technology. Also, DTs will bridge the virtual and real-world boundary, create an intelligent, humanized, and inclusive ubiquitous intelligent learning space, improve learners' personalized learning, and promote learners' overall development of cognition, skills, emotion, and body and mind.

Therefore, this article optimizes the vocal music pedagogy in higher instructions through DTs and Big Data Analytics (BDA) technologies to improve the learning efficiency of music majors. Consequently, it finds that DTs technology can build a platform connecting real teaching space and virtual teaching space. The DTs platform covers such technologies as online learning feature analysis and virtual-real teaching space fusion analysis. This article explores the online immersive teaching process design and technology application of the DTs platform from teaching and technological aspects. The advantage of this article is to explore the design and technical application of the online immersive teaching process of the DTs platform from two aspects of teaching and technology. More precisely, the DTs platform is the teaching data collection and management based on hybrid platform, teaching data analysis and modeling based on multidimensional analysis, data application based on precision teaching and precision management, and online immersive teaching experience based on Augmented Reality (AR) technology. Then, it designs its teaching process. The aim is to promote the formation of digital and intelligent classrooms and promote the innovative application of digital intelligence integration in teaching through multisource data fusion, virtual and real fusion mapping, and teaching service fusion optimization of DTs platforms.

This article first summarizes the application of DTs, BDA, and DL technology in music education. Then, it constructs an online immersive teaching system using DTs technology and analyzes the system performance by comparing the proposed system with other literature methods to point out the advantages of the proposed system. Finally, the future research direction is put forward. The innovation of this article is to construct a DTs-driven collaborative inquiry hybrid learning model under the guidance of reflective practice theory, experiential learning theory, and flipped classroom learning model. The organizational structure of the teaching platform designed by DTs technology is shown in Figure 1.

## 2. Construction of Online Immersive Education System Based on DTs

### 2.1. Application of DTs Technology in the Immersive Education System

The concept of big data was first proposed jointly by many Internet companies in the United States. Compared with traditional data, big data features large quantity, miscellaneousness, fast input and processing speed, and low data value density.  Figure 2 illustrates the big data system architecture:

DTs technology first shows itself in the 21st-century advanced manufacturing industry. It is a new concept of physical information integration. The purpose is to build a [12] simulation model of all physical, multiscale, super real, and dynamic information in the information space based on the computer-constructed potential physical and actual products. It can build an integrated physical, multiscale, ultrareal, and dynamic simulation model. Users can simulate, diagnose, predict, and monitor the manufacturing formation process, application working state, and behavior of the physical entity of the product in the real environment [13, 14].  Figure 3 displays the DTs architecture:

### 2.2. Design and Technical Analysis of Online Immersive Teaching Process

The learning environment is the learning space or place of learners. It combines various tools, resources, teacher support, and a psychological environment. It can encourage learners to explore, cooperate, interact, or solve problems with groups. Based on DTs technology, higher educational objectives, and mixed learning mode, this section constructs a collaborative inquiry learning environment driven by DTs. As drafted in Figure 4, the physics learning environment is the main place for learners to practice, experience, and interact, including classrooms, museums, and learning communities. The physical learning environment uses the twin BDA system and DTs learning environment to carry out real-time information synchronization, interactive operation, and real virtual symbiosis. Learners can realize the state observation and mutual operation of the virtual and real environment. Cloud services mainly use AI, Natural Language Processing (NLP), learning analysis, Data Mining (DM), and other technologies to process data information. Meanwhile, learners can repeatedly carry out learning activities, such as practical operation, hypothesis testing, and scheme improvement in the DTs learning environment. The intelligent brain will continue to provide suggestions for learners through the twin BDA system and constantly iterate and optimize the experimental scheme. Based on the recent related works, this article applies the DTs technology to college VME and constructs a DTs platform. The digital classroom is an online virtual teaching space enabled by DTs technologies. In particular, the DTs-enabled digital system can map the real teaching space to virtual teaching space through collaborative interaction to realize a VR integrated complex Online Teaching Platform (OTP) [15, 16]. The OTP involves online learning feature analysis technology and VR teaching space integration and analysis. Online learning feature analysis technology combines students' focus and self-discipline (virtual) with teachers' teaching resources (real). It combines students' cognitive level and growth process (virtual) with teachers' personalized guidance scheme (real) and interacts with students' technical level and understanding ability (virtual) with the key points and methods of classroom teaching (real). In this way, it truly realizes the accurate teaching and management of the whole process of online education [17, 18]. Figure 4 demonstrates the structure of the DTs platform.

The high-performance Sensor Data Acquisition (SDA) module first collects, calculates, and analyzes the students' physical signs and language features through wearables and emotion calculation model. Then, students' facial expression is captured by the cameras on the computer and mobile phone, together with body and other data information. Finally, students' learning feature data are comprehensively collected and analyzed using QS methods and other tools. High-performance SDA is the core technology of the data support layer. It can intelligently “read and write” the real teaching space through the Intelligent Sensing System (ISS), thereby realizing the DTs “nervous system” [19, 20]. In terms of online teaching data management, distributed Cloud Server (CS) storage technology provides Technical Support (TS) for data storage and management. Its efficient storage and data retrieval structure provide an important guarantee for the storage and rapid extraction of massive heterogeneous historical data. The massive multisource historical operation data also provide rich sample information for the modeling, calculation, and simulation layer, fully realize the surreal characteristics of the DTs platform, and construct a data management system throughout the whole Life Cycle (LC). The data support layer is essentially a data acquisition system based on the global stereo perception system, which realizes the omnidirectional, stereo, in-depth acquisition of teaching data [21, 22].

This article takes the vocal music pedagogy as the experimental course to analyze the online immersive teaching process design and technology application. The experimental course adopts the online immersive teaching mode and mainly uses the online learning feature analysis technology and virtual-real space fusion technology to design the teaching process [23, 24]. The online learning feature analysis technology analyzes students' online learning features and provides appropriate learning support. Virtual-real space fusion technology makes up for the boundary between the virtual-real world and improves learners' experience [25, 26]. Therefore, the overall teaching process design contains two main technical lines: online learning feature analysis and virtual-real teaching space fusion analysis. The teaching process design of the system is shown in Figure 5, and the mapping, mirroring. The collaborative operation framework of real teaching space and virtual teaching space is illustrated in Figure 6.

### 2.3. Vocal Music Feature Extraction Technology

Music feature extraction is the most important content in the evaluation system. The accuracy and scientificity of music feature extraction determine the accuracy of system signal recognition and the objectivity of evaluation results. Therefore, it is necessary to analyze music feature extraction systematically. In particular, music feature recognition is a process of transforming music materials into electronic signals. The basis of recognition is the collection of music features. This article selects four pianos and divides them into different systems, adopts different playing methods, and strengths and includes each sound region. Fourier Transform changes the collected music information to obtain the time-domain waveform and frequency-domain waveform of different music. The following equation expresses the Fourier Transform, and Figure 7 plots the extracted waveform:

(1) $$\begin{array}{c} u\left(x,t\right)=\frac{8v_{0}\delta }{\pi^{2}a}\sum_{n=1}^{\infty }\frac{1}{n}\frac{1}{1-\left(4\delta^{2}n^{2}/l^{2}\right)}\sin\frac{n\pi x_{0}}{l}\cos\frac{n\pi \;d}{l}\times \;\sin\frac{n\pi at}{l}\sin\frac{n\pi x}{l}. \end{array}$$

In equation (1), *v*_0_ is the initial motion speed of the string. *a* represents the motion acceleration. *t* and *l* are the vibration time and the chord length, respectively. *δ* denotes the half-width of the strike.

Analyzing the waveform diagram in Figure 7 proves a particular gap between the extracted music features and the actual value, so electronic music and the actual audio do not match completely. Therefore, it is necessary to process the extracted waveform to make it closer to the real value. According to relevant research, the pitch of the piano depends on the size of the fundamental frequency, and the piano's timbre depends on the size of the frequency doubling. The piano's timbre is affected by the waveform within the first five peaks in the extracted spectrum and the relative size between the five peaks. Therefore, the extraction equation must be revised again into equation (2) by considering the influencing factors of the waveform. Then, the extracted waveform is modified according to the correction equation (2), and Figure 7 is modified into Figure 8 accordingly:

(2) $$\begin{array}{c} S\left(\omega \right)=\left\{\begin{array}{c} A\frac{\alpha_{1}}{\alpha_{1}^{2}+{\left(\omega -\omega_{t}\right)}^{2}}\omega_{t}-\alpha_{1},\omega ,\omega_{t}+\alpha_{1}\\ A\frac{2}{|\omega -\omega_{t}|}other \end{array}\right). \end{array}$$

In equation (2), *S*(*ω*) is the modified vibration amplitude. *α*_1_ indicates the parameter of adjusting the waveform curve near the waveform peak. *A* represents the amplitude. *ω*_*t*_ stands for a specified audio frequency or frequency doubling.

### 2.4. Teaching Data Collection and Management Based on the Hybrid Platform

Before collecting and managing online learning features, the first step is image acquisition and recognition. Online classes generally use multiple technologies to collect students' online feature data. Image feature acquisition is completed jointly by the camera and Facial Expression Recognition (FER) and limb behavior recognition technology. Students are asked to turn on the camera first during a teaching in this article. Then, the camera is used to take pictures regularly. Finally, the Convolution Neural Networks (CNN) in DL is used for students' FER and limb behavior recognition, and BackPropagation Neural Network (BPNN) is used for classification. There are many network models in the field of DL image recognition. Model performance might vary on different datasets or even on the same set [27, 28]. Therefore, this article studies the most representative DL models: VGG Net and GoogleNet. It analyzes them from multiple aspects and improves and designs a recognition model.

VGG Net is a network model proposed by the Visual Geometry Group of Oxford University in 2014 and has achieved second place in ILSVRC2014, reducing the Top-5 Error Rate (ER) to 7.3%. The main structure of VGG Net is displayed in Table 1.

Google Net was also proposed in 2014. It is the champion of ILSVRC 2014. Its most prominent feature is introducing a network structure to improve the network's computing Resource Utilization Rate (RUR). While the depth and width of the network increase, the calculation budget remains unchanged [29, 30].  Figure 9 manifests the structure of inception [31, 32].

The designed model includes an input layer, five convolution layers, four inception modules, an average pooling layer, a full connection layer, and an output layer. The input layer inputs a 448*∗*448 RGB image different from the Google Net because large images can retain more information and have a higher definition, conducive to Feature Extraction (FE). The first layer convolution Conv1 carries out FE through 128 convolution kernels with a channel size of 3*∗*3 in step size of 2. The padding method adopts “same” to keep the image size after convolution unchanged. In contrast, the step size of 2 can reduce the image size to half, reduce the feature dimension, and then carry out nonlinear activation through ReLU Activation Function (AF). Conv1 output is 224*∗*224, and the dimension is 128 channels. The first pooling layer, Pool1, follows the first convolution layer. The window size of the pooling layer is 2 *∗* 2, the step size is also 2, and the output is half the size of the input, i.e., 112*∗*112. The dimensions remain the same. Generally speaking, the CNN model is a convolution layer followed by a pooling layer. The same is true for the proposed model. Conv2, Pool2, Conv3, and Pool3 are consistent with the previous Conv1 and Pool to extract features through multiple convolutions and pooling processes. But the parameters of these layers are slightly different. Conv4 is followed by a layer of Conv5 for FE and by Pool4 for dimension reduction. After Pool4, inspired by Google Net, four inception structures are designed to extract features. After the last inception module, a layer of pool8 is connected to compress the features further. The last layer is the final output layer, and the output size is 1*∗*1*∗*64. The specific parameters of each layer are demonstrated in Table 2.

### 2.5. Teaching Data Analysis and Modeling Based on Multidimensional Analysis

Multidimensional data analysis in the vocal music pedagogy course is mainly used in online learning feature analysis and mining. In contrast, multidimensional data modeling is used for virtual-real teaching space fusion simulation and modeling. In the online learning feature analysis and mining, the experimental course creates the student portrait model through data feature recognition, data analysis, and data association analysis. Multidimensional modeling in the experimental course includes real-time modeling technology, virtual simulation technology, and virtual-real fusion technology. Specifically, real-time modeling technology is the basis of virtual simulation technology and virtual-real fusion. Combining real-time modeling technology with virtual simulation technology can be used for big data visual analysis of virtual-real teaching space based on AI technology. Combining real-time modeling technology and virtual-real fusion technology mainly uses big data analysis, mining, and modeling technology. It analyzes the association rules of various algorithms for the association of virtual and real teaching space, deeply analyzes the relationship between virtual and real teaching space, and promotes the integration of virtual-real teaching space around this relationship. The construction of digital teaching space is mainly based on the modeling of real teaching space, but the modeling is based on the relationship between virtual space and real space. Therefore, according to the basic principles of Educology and Psychology, this articles marks the different elements in the real teaching space by extracting the keywords or features of the real teaching space and then constructs the relevant feature model via Machine Learning (ML) approaches. For example, big data text mining is used to analyze and visualize the structure of textbook content; the matrix correlation algorithm is used to construct the correlation between virtual-real teaching space elements.

### 2.6. Experimental Environment Configuration and Dataset

Table 3 shows the parameter configuration of experimental hardware and software.

Then, the accuracy is used to evaluate the model's performance, as calculated by the following equation:

(3) $$\begin{array}{c} Accura\text{cy}=\frac{TP+TN}{TP+FN+FP+TN}. \end{array}$$

In equation (3), *TP* means that a positive sample is classified as positive, and *TN* indicates that a negative sample is classified as negative. *FP* suggests that a negative sample is classified as positive, and *FN* implies that a positive sample is classified as negative.

The proposed network model uses JAFFE dataset for training and testing, in which there are 213 images. Ten Japanese female students are selected, and each of them makes seven expressions, including anger, disgust, fear, happiness, sadness, surprise, and neutrality.

## 3. Experimental Results and Analysis

### 3.1. Algorithm Performance Analysis

Optimization algorithms might have different effects on the proposed model. Hence, this section selects Stochastic Gradient Descent (SGD), Root Mean Square Prop (RMSProp), and Adaptive Motion Estimation (Adam) to compare them with the proposed model. According to the previous analysis, the model AF is ReLU, the number of convolution kernels is set as the default value, and the number of training iteration steps is uniformly set to 8,000 steps. The results are plotted in Figure 10.

Figure 10 indicates that the results of several optimization methods are similar. The difference is that the convergence speed of the Adam method is faster than that of the RMSPROP. The speed of SGD may be faster, but the accuracy is unstable, especially in the middle, the accuracy fluctuates dramatically. Therefore, after careful consideration, this article selects the Adam algorithm as the optimization algorithm.

Subsequently, it verifies the superiority of the proposed model by comparing its FER results with that of the classical target detection model.  Figure 11 reveals a comprehensive comparison in terms of factors, such as accuracy and loss magnitude.

Figure 11 corroborates that after 10,000 steps of iterative training, the recognition accuracy of the proposed model reaches the highest (99.08%). In contrast, the accuracy of VGG Net and Google Net is not low, reaching more than 94%. However, the proposed model has significantly more advantages in training time and network depth. The comparison between VGG Net and Google Net implies that the deeper the network is, the better the recognition effect is in most cases. The proposed model improves the recognition accuracy and reduces the training time by optimizing the network structure, reasonably setting parameters, selecting the AF, and adding dropout. Hence, the proposed model has certain advantages.

Further, this section utilizes 15,000 image data from the student expression set to verify multiple models. The results are shown in Figure 12, which proves that the proposed model has an average recognition accuracy of 85%. It can be applied to the students' FER and body movements recognition. Figure 12 illuminates the model performance test.

## 4. System Performance Comparison Test

Figure 13 depicts the feedback results of students to the teaching system.

Figure 13(a) implies no noticeable fluctuation in the active and passive interaction curve of the traditional VME system. Thus, the conventional VME system is not interactive, has poor ability to actively feedback information, and has no positive feedback to users' questions. The test results of the proposed VME system are shown in Figure 13(b). The time of information submission and feedback in the VME system is relatively close, and there is little change in the whole experimental process. The active and passive interaction curves fluctuate greatly, proving that the proposed VME system has more frequent interaction. The teaching information can get real-time and active feedback. Hence, the proposed system can better stimulate students' learning desire.

### 4.1. Student Achievement Prediction and Analysis Experiment

Figure 14 shows the students' actual scores of the Vocal Music Subject and the BPNN-predicted and Genetic Neural Network (GNN)-predicted scores for ten students after using the proposed system.

As detailed in Figure 14, for student 1, the actual score of Vocal Music Subject is 74 points. BPNN and GNN predict the score to be 67 and 69 points, respectively. Comparing the student performance predicted by BPNN and GNN with the real performance corroborates that the student performance predicted by the GNN model is closer to the real performance and has less prediction error. Overall, the proposed system can improve students' performance to some extent.

### 4.2. Experimental Comparison and Discussion

The experiment adopts the quasiexperimental research method. The experimental group and control group both consist of 24 respondents. The pretest shows that respondents have no significant differences in learning attitude, motivation, and innovative thinking. Then, different teaching methods are implemented for the two groups. The experimental group learns by combining text, picture, and DTs system, while the control group learns by combining text and picture. After teaching implementation, the two groups of students will be posttested.  Table 4 presents the comparison of experimental results.

Firstly, in the dimension of learning attitude, there is no significant difference between the students who use the proposed method and those who use the literature method proposed by Roy et al. [33]. Learners believe that the relevant learning contents of music knowledge are important and valuable. They can actively collect learning materials, but this is not closely related to learning methods. On the other hand, students believe that learning attitude is more related to teaching style, learning interest, and internal motivation. The value of knowledge itself is closely related to learners' needs, and the influence of teaching methods on students is not significant. Secondly, there are significant differences in learning motivation between students who use the proposed methods and those who use the method proposed by Roy et al. This indicates that the learning motivation of the two groups of students is not significantly affected by different teaching methods. Overall, under the two learning methods of the DTs system or learning based on words and pictures, learners fail to enhance their internal and external motivation. The two systems only offer students learning methods rather than incentives to stimulate their internal and external needs. Thirdly, there are significant differences in self-learning efficacy between students who use the proposed methods and those who use the methods proposed by Roy et al. Therefore, using the DTs system enhances learner confidence in understanding, observing, and mastering relevant knowledge. On the contrary, learners relying on text and picture learning face great cognitive pressure.

## 5. Conclusions

As a representative product of computer technology in the era of AI, DTs classroom is reshaping the teaching perception and experience mode and changing the way of thinking to solve problems. It realizes the subversive transformation of online teaching towards data-driven, field quantification, and data visualization modes. Meanwhile, the DTs platform is an important means of online immersive education innovation in education informatization. It is also a crucial innovative application of AI technology in online education reform. Accordingly, this article preliminarily constructs an online immersive education system for VEM based on the DTs platform and uses the DTs and BDA technology to design the specific teaching process. The experimental results show that the constructed NN has the highest recognition accuracy of 99.07% on the student action and expression dataset. When tested with the image data taken by the research experiment, the highest accuracy is 89%, with an average of more than 85%. Further, the constructed VME system has shown frequent teacher-student interaction, and the teaching information can get real-time and active feedback. Thus, the constructed system can better stimulate students' desire to learn music. Lastly, the design and implementation of the teaching system are completed in the experimental environment, yet, in the practical application of academia, there is uncertainty in the teaching and learning ability of students and teachers, which requires the system to have high performance and efficiency. At the same time, the evaluation of the system hard index is carried out on the simulated data. In practical application, whether the proposed method can meet the system requirements and produce satisfactory benefits must be considered in detail. The future work will further extend the experimental time in applying DTs education to observe its impact on other aspects of students. Additionally, the government, enterprises, and schools need to work together to create a fully functional DTs learning space for learners and build a future DTs learning world, including DTs laboratories, DTs cities, and DTs factories.

## Figures and Tables

**Figure 1:** Organizational structure of teaching platform.

**Figure 2:** Big data system architecture.

**Figure 3:** DTs framework.

**Figure 4:** DTs platform structure.

**Figure 5:** Systematic teaching process.

**Figure 6:** Mapping, mirroring, and cooperative operation framework of real teaching space and virtual teaching space.

**Figure 7:** Waveform before processing. (a) Time-domain waveform; (b) frequency-domain waveform.

**Figure 8:** Processed waveform. (a) Frequency-domain waveform; (b) local waveform.

**Figure 9:** Inception structure.

**Figure 10:** Comparison of different optimization algorithms. (a) The first test results; (b) the second test results.

**Figure 11:** Algorithm performance comparison. (a) The first test results; (b) the second test results.

**Figure 12:** Model performance test.

**Figure 13:** Test results of teaching system. (a) System test results before improvement; (b) system test results after improvement.

**Figure 14:** Student's real score broken line, BPNN prediction broken line, and GNN prediction broken line. (a) The first test structure; (b) the second test results.

**Table 1:** VGGNet structure.

A	A-LRN	B	C	D	E
11 weight layers	11 weight	13 weight	16 weight	16 weight	19 weight layers
	Layers	Layers	Layers	Layers	
Input (224 × 224 RGB image)					
conv3-64	conv3-64	conv3-64	conv3-64	conv3-64	conv3-64
	LRN	conv3-64	conv3-64	conv3-64	conv3-64
Max pool					
conv3-128	conv3-128	conv3-128	conv3-128	conv3-128	conv3-128
		conv3-128	conv3-128	conv3-128	conv3-128
Max pool					
conv3-256	conv3-256	conv3-256	conv3-256	conv3-256	conv3-256
conv3-256	conv3-256	conv3-256	conv3-256	conv3-256	conv3-256
			Convl-256	conv3-256	conv3-256
					conv3-256
Max pool					
conv3-512conv3-512	conv3-512	conv3-512	conv3-512	conv3-512	conv3-512
	conv3-512	conv3-512	conv3-512	conv3-512	conv3-512
			Convl-512	conv3-512	conv3-512
					conv3-512
Max pool					
conv3-512conv3-512	conv3-512	conv3-512	conv3-512	conv3-512	conv3-512
	conv3-512	conv3-512	conv3-512	conv3-512	conv3-512
			Convl-512	conv3-512	conv3-512
					conv3-512
Max pool					
FC-4096					
FC-4096					
FC-1000					
SoftMax					

**Table 2:** Network structure parameter.

Type	Convolution kernel size/Step size	Number of convolution kernels	Output
Input	—	—	448*∗*448*∗*3
Conv1	3*∗*3/2	128	224*∗*224*∗*128
Pool1	2*∗*2/2	—	112*∗*112*∗*128
Conv2	3*∗*3/1	256	112*∗*112*∗*256
Pool2	3*∗*3/1	—	56*∗*56*∗*256
Conv3	3*∗*3/1	256	56*∗*56*∗*256
Pool3	3*∗*3/2	—	28*∗*28*∗*256
Conv4	1*∗*1/1	128	28*∗*28*∗*128
Conv5	3*∗*3/1	128	28*∗*28*∗*128
Pool4	3*∗*3/2	—	14*∗*14*∗*128
Inception1	—	64/64, 96/16, 32/32	14*∗*14*∗*224
Pool5	3*∗*3/2	—	7*∗*7*∗*224
Inception2	—	64/64, 96/16, 32/32	7*∗*7*∗*224
Pool6	3*∗*3/2	—	4*∗*4*∗*224
Inception3	—	64/64, 96/16, 32/32	4*∗*4*∗*224
Pool7	2*∗*2/1	—	2*∗*2*∗*224
Inception4	—	64/64, 96/16, 32/32	2*∗*2*∗*224
Pool8	2*∗*2/1	—	1*∗*1*∗*224
Output	1*∗*1/1	—	1*∗*1*∗*64

**Table 3:** Experimental environment configuration.

Hardware platform parameters	Software environment parameters
Intel core I7-6700K quad core eight thread CPU	Ubuntu 16.04
Nvidia GTX 2060 GPU	CuDNN 7.4, CUDA 9.1

**Table 4:** Comparison of experimental results.

Analysis dimension	Measurement	Mean value	Standard deviation	T	*P*
Learning attitude	Proposed method	11.67	2.12	1.804	0.078
	Literature method proposed by Roy et al. [33]	10.42	2.65		

Learning motivation	Proposed method	11.5	2.22	1.334	0.189
	Literature method proposed by Roy et al. [33]	10.67	2.09		

Self-learning efficacy	Proposed method	10.71	2.26	2.125	0.039
	Literature method proposed by Roy et al. [33]	9.21	1.62		

## Data Availability

The raw data supporting the conclusions of this article will be made available by the authors without undue reservation.
